This article has been retracted.

# Regulation of Proapoptotic Mammalian ste20–Like Kinase MST2 by the IGF1-Akt Pathway

**DOI:** 10.1371/journal.pone.0009616

**Published:** 2010-03-09

**Authors:** Donghwa Kim, Shaokun Shu, Marc D. Coppola, Satoshi Kaneko, Zeng-qiang Yuan, Jin Q. Cheng

**Affiliations:** Department of Molecular Oncology, H. Lee Moffitt Cancer Center and Research Institute, Tampa, Florida, United States of America; University of Texas MD Anderson Cancer Center, United States of America

## Abstract

**Background:**

Hippo, a *Drosophila* serine/threonine kinase, promotes apoptosis and restricts cell growth and proliferation. Its mammalian homolog MST2 has been shown to play similar role and be regulated by Raf-1 via a kinase-independent mechanism and by RASSF family proteins through forming complex with MST2. However, regulation of MST2 by cell survival signal remains largely unknown.

**Methodology/Principal Findings:**

Using immunoblotting, *in vitro* kinase and *in vivo* labeling assays, we show that IGF1 inhibits MST2 cleavage and activation induced by DNA damage through the phosphatidylinosotol 3-kinase (PI3K)/Akt pathway. Akt phosphorylates a highly conserved threonine-117 residue of MST2 *in vitro* and *in vivo,* which leads to inhibition of MST2 cleavage, nuclear translocation, autophosphorylation-Thr180 and kinase activity. As a result, MST2 proapoptotic and growth arrest function was significantly reduced. Further, inverse correlation between pMST2-T117/pAkt and pMST2-T180 was observed in human breast tumors.

**Conclusions/Significance:**

Our findings demonstrate for the first time that extracellular cell survival signal IGF1 regulates MST2 and that Akt is a key upstream regulator of MST2.

## Introduction

MST2 and its close homologue MST1 are members of the germinal center kinase group II (GCK II) family of mitogen-activated protein kinase (MAPK)–related kinases that includes the more distantly related kinases MST3, MST4, LOK, SOK, and SLK. Unlike other members, MST1 and MST2 contain a Ste20-related kinase catalytic domain in the N-terminal region followed by a noncatalytic tail that contains an autoinhibitory domain, a dimerization domain, and two nuclear export sequences at the COOH terminus [1], [2], [3]. It has been shown that the noncatalytic tail is cleaved by caspase upon various apoptotic stimuli [4], [5], [6]. Ectopic expression of MST1/2 induces striking morphological changes characteristic of apoptosis in both nucleus and cytoplasm. During the execution phase of apoptosis in mammalian cells induced by proapoptotic stimuli, MST1 and MST2 are activated by caspase cleavage and subsequently translocated to the nucleus. In the case of MST1, this leads to a constitutive phosphorylation of H2B, resulting in nuclear DNA fragmentation [7]. It has been shown that the protective function of the Raf1 (including kinase-dead Raf-1) against apoptosis involves the inhibition of MST2 activity by direct sequestration and inhibition of MST2 activation [8], [9]. In addition, RASSF (Ras association domain family) proteins RASSF1A and RASSF5 have been demonstrated to bind MST1 [10], [11], [12]. RASSF1A also releases MST2 from the inhibitory effect of Raf-1[13]. RASSF1A also releases MST2 from the inhibitory effect of Raf-1 [13]. Ultimately, RASSF1A and RASSF5 activate NDR1, NDR2, and LATS1 to induce apoptosis [13], [14], [15], [16]. These findings suggest that RASSF1A and RASSF5 stimulate MST signaling. A recent study shows that RASSF6 interacts with MST2 and inhibits MST2 activity. However, RASSF6 caused apoptosis when released from activated MST2 in a manner dependent on WW45 [17]. These findings suggest that activation of MST2 causes apoptosis through the canonical pathway, as well as through a RASSF6-mediated pathway [17].

In *Drosophila*, Hippo, a homolog of mammalian MST2, restricts cell growth and cell proliferation and promotes cell death by interaction with the tumor suppressors Salvador (Sav)/WW45 and Warts (Wts)/Lats1/Lats2, which result in inhibition of transcription and/or degradation of cyclin E and DIAPs [18], [19], through phosphorylation of Yorkie, which is the *Drosophila* ortholog of the mammalian transcription co-activator yes-associated protein (YAP) [20]. YAP and Yorkie have recently been shown to be negatively regulated by the Hippo/MST pathway and play an important role in mediating cell contact inhibition, organ size and tumorigenesis [21], [22].

Accumulated evidence shows that Akt and its downstream targets constitute a major cell survival pathway. Akt inhibits the programmed cell death in a number of cell types induced by a variety of stimuli through regulation of down stream molecules [23], [24]. Akt phosphorylates BAD on serine 136, which promotes the association of BAD a pro-apoptotic protein in Bcl-2 family, with 14-3-3 proteins in the cytosol, thus inactivating its pro-apoptotic function [25]. In addition, Akt reduces the transcription of a subset of pro-apoptotic genes by phosphorylation of Forkhead transcription factors, which causes their nuclear exclusion and inactivation [26], including FOXO1, FOXO3a, and FOXO4 and the phosphorylation by Akt negatively regulates FOXO activity by relocalizing FOXO from nucleus to the cytoplasm, where it is sequestered away from target genes through interacting with 14-3-3 [27]. In addition, several pro-apoptotic and anti-apoptotic proteins are also phosphorylated by Akt, including ASK1 [28], XAIP [24], Par-4 [29], BAX [30], [31], HtrA2 [32], which leads to direct activation of cell survival pathway.

A previous study showed that EGF stimulation caused a drop of MST1 kinase activity [33]. However, the regulation of MST2/Hippo by cell survival signaling remains largely unknown. In this report, we demonstrate that MST2 is inhibited by IGF1 through the PI3K/Akt pathway. Akt phosphorylates MST2 at Thr117 *in vitro* and *in vivo*, which leads to inhibition of MST2 cleavage and kinase activity as well as nuclear translocation. Furthermore, Akt activation is inversely correlated with autophosphorylation of MST2-T180 but paralleled with MST2-T117 phosphorylation in breast tumors. Collectively, our findings suggest that MST2 is a *bona fide* substrate of Akt and that Akt could play a critical role in regulation of the Hippo/MST2 pathway.

## Materials and Methods

### Reagents, Cell Culture and Breast Tumor Specimens

Stauroporine, LY294002 were obtained from Sigma (St. Louis, MO). DMEM and fetal bovine serum were purchased from Invitrogen Co. (Grand Island, NY). Anti-MST2 (#3952), -pMST2-Thr180 (#3681), -Akt (#9272), -pAkt-Ser473 (#9271), -actin (#4967) and -cleaved PARP (#9541 and #9544) antibodies were from the Cell Signaling Technology (Beverly, MA). Anti-GFP antibody was purchased from Santa Cruz Biotechnology (Santa Cruz, CA). COS7 and human embryonic kidney (HEK) 293 cells were purchased from The American Type Culture Collection (ATCC; Manassas, VA) and cultured at 37°C and 5% CO2 in DMEM supplemented with 10% fetal bovine serum. Eighty primary human breast cancer specimens were obtained from patients who underwent surgery at H. Lee Moffitt Cancer Center and approved by Institutional Review Board. Each sample contains at least 80% tumor cells, confirmed by microscopic examination.

### Expression Constructs

Flag-tagged MST2 was created by PCR amplification of human Fetal Marathon-Ready cDNA (Clontech). The PCR products were cloned to p3XFLAG-CMV-10 vector (Sigma) at *Eco*RI-*Bam*HI sites. MST2 specific primers are: ccggaattcatggagcagccgccggcg (5′primer), and cgcggatccaaagttttgctgccttct (3′primer). Flag-MST2-T117A and Flag-MST2-T117D were produced with mutagenesis kit (Stratagene) using wild-type MST2 as template. Wild type MST2 and mutant MST2 were also cloned to pEGFP-C1 (Clontech) at *Eco*RI-*Bam*HI sites. GST-MST2 and GST-MST2-T117A were created by PCR amplification of 150 nucleotide fragment (a.a. 100–150) which include T117 and T117A sites using Flag-MST2-T117A and Flag-MST2-T117D as templates. The fragments were cloned to pGEX-4.1 vector at *Bam*HI-*EcoR*I sites. The MST2 plasmids were confirmed by DNA sequencing. Akt expression constructs were previously described [32].

### Immunoprecipitation, Immunoblotting and *In Vitro* Kinase Assay

Immunoprecipitation and immunoblotting were performed as previously described [24]. The immunoprecipitates were subjected to Western blotting analysis or *in vitro* kinase assay. Protein kinase assays were performed as previously described [34]. Briefly, reactions were carried out in the presence of 10 µCi of [γ-32P] ATP and 3 µM cold ATP in 30 µl buffer containing 20 mM Hepes (pH 7.4), 10 mM MgCl_2_, 10 mM MnCl_2_, and 1 mM dithiothreitol using myelin basic protein (MBP) as substrate. After incubation at room temperature for 30 min the reaction was stopped by adding protein loading buffer and proteins were separated on SDS-PAGE gels. Each experiment was repeated three times and the relative amounts of incorporated radioactivity were determined by autoradiography and quantified with a Phosphoimager (Molecular Dynamics).

### *In Vivo* [^32^P] Pi Labeling

COS7 cells were co-transfected with kinase-dead Flag-MST2 and constitutively active Akt. Following 48 h incubation, cells were labeled with [^32^P] Pi (0.5 mCi/ml) in phosphate- and serum-free DMEM medium for 4 h and then lysed. Cell lysates were subjected to immunoprecipitation with anti-Flag antibody. The immunoprecipitates were separated by 7.5% SDS-PAGE and transferred to membranes. The phosphorylated MST2 band was visualized by autoradiography.

### Cell Death Assay, TUNEL Assay, Caspase3/7 Assay

Cells were seeded into 60-mm dishes and grown in DMEM supplemented with 10% FBS for 24h, treated with STS (30 µM). Apoptosis was determined by Tunel assay using an in situ cell death detection kit (Boehringer Mannheim, Indianapolis, IN) and caspase 3/7 assay kit (Promega). These experiments were performed three times in triplicate.

## Results

### IGF1 Inhibits MST2 through the PI3K/Akt Pathway and Akt Regulates MST2 Activation

Since MST2 is cleaved and activated upon apoptotic stimuli and is required for DNA damage-induced apoptosis in different types of cells, we initially examined if extracellular cell survival signal regulates MST2 cleavage and activation. COS7 cells were treated with staurosporine (STS; 1 µM) together with and without IGF1 for 2 h. Consistent with previous studies, STS alone induces MST2 cleavage and autophosphorylation of Thr180, an indicator of MST2 activation, as well as apoptosis. However, addition of IGF1 largely reduced STS effect towards MST2. PI3K inhibitor LY294002 inhibited the IGF1 action (Figure 1a). Further, LY294002 and Akt inhibitor API-2 [35] were able to induce MST2 activation and cleavage, which is inhibited by pan-caspase inhibitor Z-VAD (Figure 1b). These results imply that STS-induced MST2 cleavage and activation are inhibited by IGF1 through the PI3K/Akt pathway.

**Figure 1:** IGF1/PI3K/Akt inhibits MST2 cleavage, activation and MST2-induced cell death. (a) IGF1 inhibits MST2 through the PI3K/Akt pathway. Top panel is domain structure of MST2. DELD is a caspase cleavage motif and NES stands for nuclear export signal. Middle panels are immunoblots of COS7 cells, which were treated with IGF1 (50 µM) or/and LY294002 (20 µM) for 30 min prior to exposure to STS (1 µM) for 1 h, with indicated antibodies. Bottom panel shows the apoptosis measured with Tunel assay in three experiments in triplicate. (b) Inhibitors of PI3K (LY294002) and Akt (API-2) activate MST2. After treatment with indicated compounds for 3 h, COS7 cells were subjected to immunoblotting with indicated antibodies (upper panels) and apoptosis analysis (bottom). (c) Reconstitution of Akt in Akt1-null MEFs reduces MST2 activation induced by STS. Akt1-knockout MEFs were infected with adenovirus expressing Akt and then treated with 0.2 µM STS for 1h. Immunoblotting (upper) and apoptosis (bottom) analyses were performed as described above. (d) Knockdown of Akt enhances doxorubicin-activated MST2. MDA-MB-468 cells were transfected/treated with Akt/shRNA together with or without doxorubicin, and then subjected to immunoblotting (upper) and Tunel (bottom) analyses. (e) and (f) Constitutively active (Ac) Akt inhibits but dominant-negative (DN) Akt induces MST2 activation. COS7 cells were transfected with indicated plasmids. Following 48 h of incubation, cells were assayed for autophospho-T180 (top panel of e) and *in vitro* MST2 kinase using MBP as substrate (top panel of f). Middle and bottom panels show expression of the transfected plasmids.

We next examined the effect of Akt on MST2 activation. Akt-knockout MEFs were infected with adenovirus expressing Akt and adenovirus vector alone as control. STS treatment at low concentration (0.2 µM) considerably induces MST2 activation and cleavage as well as apoptosis in Akt-null MEF but not Akt-reconstituted cells (Figure 1c). Moreover, knockdown of Akt1 induces MST2 activation and enhances doxorubicin-activated MST2 and apoptosis in PTEN-mutated MDA-MB-468 cells (Figure 1d). Further, ectopic expression of dominant-negative Akt induces whereas constitutively active Akt represses MST2-Thr180 autophosphorylation in COS7 cells (Figure 1e). Constitutively active Akt also inhibited the apoptosis induced by ectopic expression of MST2 in MCF10A cells (Figure S1). *In vitro* MST2 kinase activity was also inhibited by ectopic expression of wild-type and constitutively active Akt (Figure 1f).

### Akt Interacts with and Phosphorylates MST2

We next investigated whether Akt forms a complex with MST2. COS7 cells were co-transfected with HA-Akt and Flag-MST2. Co-immunoprecipitation experiments revealed that Flag-MST2 was readily detected in HA-Akt immunoprecipitates and vice versa (Figure 2a). Having demonstrated constitutively active Akt inhibition of MST2 but dominant-negative Akt activation of MST2 (Figure 1), we reasoned Akt regulation of MST2 through a kinase-dependent mechanism. Sequence analysis shows a well-conserved Akt phosphorylation consensus motif (^112^ **R**L**R**NK**T** ^117^) in a kinase domain of MST2 (Figure 2b). *In vivo* [^32^P]orthophosphate labeling and immunoblotting analysis with Akt substrate antibody revealed that constitutively active Akt induced MST2 phosphorylation (Figures 2c and 2d). Further, we created wild-type and T117A GST-MST2 (a.a. 100–150) fusion proteins which were used as substrate for *in vitro* Akt kinase assay. Figure 2e shows that Akt phosphorylates wild-type but not T117A MST2. These data suggest that MST2 is an Akt substrate.

**Figure 2:** Akt interacts with and phosphorylates MST2. (a) MST2 binds to Akt. COS7 cells were co-transfected with Flag-MST2 and HA-Akt. After 48 h of transfection, cells were lysed, immunoprecipitated with anti-Flag and detected with HA antibody (top) and vice versa (bottom). (b) Sequence alignment shows a highly conserved Akt phosphorylation consensus site of MST2 among different species. (c) and (d) Akt phosphorylates MST2 *in vivo*. COS7 cells were transfected with kinase-dead Flag-MST2 together with or without constitutively active (Ac) dominant-negative (DN) Akt. Following 36 h of transfection, cells were either labeled by [^32^P]-orthophosphate (c) or immunoprecipitated with anti-Flag antibody and immunoblotted with anti-Akt-substrate antibody (top panel of d). For *in vivo* labeled cells, immunoprecipitation was performed with anti-Flag antibody and exposed to a film (top panel of c). Middle and bottom panels show expression of the transfected plasmids. (e) Akt phosphorylates MST2-T117 *in vitro*. *In vitro* Akt kinase assay was carried out by incubation of recombinant active Akt and GST-WT-MST2 and -MST2-T117A fused proteins (top). Bottom panel is coomassie blue staining of GST-MST2 proteins.

### Akt Phosphorylates MST2-T117 *In Vivo* and the pMST2-T117 Inhibits Thr180 Autophosphorylation

To demonstrate *in vivo* phosphorylation of MST2-T117 by Akt, we generated specific phospho-MST2-T117 antibody by immunization of a rabbit with phospho-peptides (Ac-IRLRNK(pT)LIEDEIA-amide). We first characterized the specificity of this antibody. HEK293 cells were co-transfected with constitutively active HA-Akt and full-length wild-type and T117A mutant Flag-MST2. After immunoprecipitation with anti-Flag antibody, immunoblotting analysis with anti-pMST2-T117 antibody revealed that Akt phosphorylates wild-type but not T117A mutant MST2 (Figure 3a). We further showed that ectopic expression of wild-type or constitutively active Akt induced MST2-T117 phosphorylation whereas dominant negative Akt decreased the phosphorylation compared to that of the cells transfected with vector alone (Figure 3b).

**Figure 3:** Akt phosphorylates Thr117 of MST2 *in vivo* and the pMST2-T117 regulates autophospho-MST2-T180. (a) Characterization of anti-pMST-T117 antibody. HEK293 cells were transfected with constitutively active Akt and Flag-MST2 or Flag-MST2-T117A and immunoprecipitated with anti-Flag antibody. The immunoprecipitates were immunoblotted with anti-pMST2-T117 antibody (top). Middle and bottom panels show expression of the transfected plasmids. (b) Akt phosphorylates endogenous MST2-T117. Following transfection of HEK293 cells with indicated different Akt, cells were lysed and immunoblotted with anti-pMST2-T117 (top), -MST2 (panel 2), -HA (panel 3) and -actin (bottom) antibodies. (c) IGF1 induces pMST2-T117 and represses pMST2-T180. After serum starvation for 12 h, HEK293 cells were stimulated with IGF1 for 1 h and then immunoblotted with indicated antibodies. (d) Re-expression of Akt in Akt1^-/-^ MEF increases pMST2-T117 and reduces pMST2-T180 level. Akt1-null MEFs were infected with adenovirus expressing Akt or control vector and immunoblotted with indicated antibodies. (e) Knockdown of Akt decreases pMST2-T117 and increases pMST2-T180. MDA-MB-468 cells were transfected with AKT1/shRNA and control shRNA. After 72 h incubation, cells were lysed and immunoblotted with indicated antibodies. (f) Phospho-Thr117 regulates MST2 autophosphorylation of Thr180. HEK293 cells were transfected with indicated plasmids and immunoprecipitated with anti-Flag antibody. The immunoprecipitates were immunoblotted with anti-pMST2-T180 (top) and -Flag (bottom) antibodies.

In addition, serum starvation reduces whereas IGF1 induces pMST2-T117 levels (Figure 3c). Introduction of Akt into Akt-null MEFs also increases pMST2-T117 (Figure 3d). Notably, pMST2-T117 is inversely correlated with autophosphorylation of Thr180 (Figures 3c and 3d). We also observed that knockdown of Akt in MDA-MB-468 cells reduced pMST2-T117 but increased pMST2-T180 (Figure 3e). Based on these findings, we hypothesized that Akt phosphorylation of Thr117 is required for inhibition of autophosphorylation of Thr180 of MST2. To test this, we introduced Akt phosphomimetic Flag-MST2-T117D and nonphosphorylatable Flag-MST2-T117A as well as wild-type Flag-MST2 into HEK293 cells. After immunoprecipitation with Flag antibody, immunoblotting analysis revealed that antophosphorylation of MST2-T180 was detected in the cells transfected with MST2-T117A and MST2 but not with MST2-T117D (Figure 3f). Collectively, we conclude that MST2 is *bona fide* substrate of Akt and the phosphorylation of Thr117 negatively regulates pMST2-T180.

### Akt Inhibits MST2 Nuclear Translocation, Cleavage and Kinase Activity via a pThr117-Dependent Mechanism

Because the MST2 cleavage and nuclear translocation are critical steps for MST2 function and because Akt phosphorylates MST2-T117, we reasoned that Akt could inhibit MST2 nuclear translocation and that this action could depend on phosphorylation of Thr117. To this end, we created GFP-tagged wild-type MST2, Akt phosphomimetic MST2-T117D and nonphosphorylatable MST2-T117A. After transfection of COS7 cells with the various forms of GFP-MST2 together with and without constitutively active Akt, subcellular localization of GFP-MST2 was examined under a fluorescence microscope. Figure 4a shows that STS treatment induces WT-MST2 nuclear translocation which was inhibited by constitutively active Akt. Under non-DNA damage (e.g., STS) condition, constitutively active Akt also reduced approximately half of ectopically expressed wild-type MST2 nuclear translocation (Figure 4b). MST2-T117A exhibited nuclear localization whereas MST2-T117D located at cytoplasm. Expression of constitutively active Akt had no effect on subcellular localization of MST2-T117A and MST2-T117D (Figure 4b).

**Figure 4:** Akt phosphorylation of Thr117 reduces MST2 nuclear translocation and activation. (a) and (b), Akt inhibits wild-type MST2 nuclear translocation but has no effects on MST2-T117A and MST2-T117D. Panel (a) shows that STS-induced MST2 nuclear translocation was inhibited by Akt. COS7 cells were transfected with GFP-MST2 together with and without constitutively active Akt. After STS treatment for 2 h, cellular distribution of MST2 was examined (top) and quantified (bottom) under fluorescent microscopy. In panel b, COS7 cells were transfected with different forms of GFP-MST2 together with and without constitutively active Akt. After 36 h incubation, cells were examined and quantified for the nuclear MST2. The experiments were repeated for three times and 200 cells/transfection were examined. (c) Phospho-Thr117 reduces MST2 cleavage and kinase activity. COS7 cells were transfected with indicated plasmids. Following treatment with and without STS, cells were subjected to immunoblotting (top) and immunoprecipitation with anti-Flag antibody. The immunoprecipitates were subjected to *in vitro* MST2 kinase assay using MBP as substrate (bottom). (d) Akt failed to inhibit STS-induced MST2-T117A cleavage and kinase activity. COS7 cells were transfected/treated with indicated plasmids and reagent and then subjected to Western blot (top) and *in vitro* MST2 kinase assay (bottom) as described above.

Having demonstrated Akt inhibition of MST2 nuclear translocation through phosphorylation of Thr117, we next examined if Akt inhibition of MST2 cleavage and kinase activity depends on phosphorylation of Thr117. After transfection with Flag-tagged wild-type and mutant MST2 together with and without constitutively active Akt, COS7 cells were treated with STS or vehicle. Immunoblotting analysis shows that STS treatment induced the cleavage of MST2-T117A and wild type MST2, but had no significant effect on the cleavage of MST2-T117D (Figure 4c). Moreover, ectopic expression of constitutively active Akt reduced STS-stimulated wild-type MST2 but not MST2-T117A cleavage (Figure 4d). We have also examined whether the Akt phosphorylation of thr-117 affects MST2 kinase activity. *In vitro* kinase assays revealed that basal kinase activity was considerably reduced in phosphomimetic MST2-T117D whereas nonphosphorylatable MST2-T117A exhibited much higher kinase activity compared to wild type MST2 in the absence or presence of STS (Figure 4c). In combination of the findings in Figure 2b, these data indicate that full-length MST2-T117A is able to translocate to the nucleus and exhibits high level of kinase activity whereas MST2-T117D remains in cytoplasm and loses its kinase activity. Further, Akt had no effect on MST2-T117A kinase activity (Figure 4d). Taken collectively, these results indicate that phosphorylation of Thr117 is required for Akt inhibition of MST2 cleavage, nuclear translocation and kinase activity.

### Phosphorylation of Thr117 Reduces MST2-Induced Apoptosis and Growth Arrest and Is Associated with pAkt in Breast Cancer

We next examined the effects of phosphorylation Thr117 on MST2-regulated cell survival and growth. Figure 5a shows that ectopic expression of MST2 and MST2-T117A in HEK293 cells induced PARP cleavage whereas MST2-T117D had no effect on PARP cleavage compared to the cell transfected with vector alone. Caspase-3/7 activity was also increased by expression of MST2 and MST2-T117A but not MST2-T117D. Moreover, constitutively active Akt reduced the effect of wild-type MST2 but had no influence on MST2-T117A and MST2-T117D (Figure 5b). Previous studies have also shown that MST2 activation inhibits cell proliferation [36]. Thus, we have performed cell proliferation assay and observed that cell growth was significantly decreased in MST2-T117A cells whereas increased in MTS2-T117D cells when compared to wild-type-MST2 and vector-transfected cells (Figure 5c). Because Akt phosphorylation of MST2-T117 inhibits autophospho-MST2-T180 (Figures 2 and 3), we also investigated whether this regulation also existed in tumor tissues. Western blot analysis was performed in 80 human primary breast carcinomas. Elevated levels of phospho-Akt were detected in 40 specimens (Figure 5d and data not shown), 33 of which exhibited high levels of phospho-MST2-T117 whereas 35 of which express low or undetectable level of phospho-MST2-T180. Notably, all 33 tumors with high levels of phospho-Akt/phospho-MST2-T117 had low phospho-MST2-T180. Statistic analysis revealed that phospho-Akt significantly links to phospho-MST2-T117 (p<0.0001) which inversely correlates with phospho-MST2-T180 (p<0.0001; Figure 5e). In addition, overall survival of the patients with elevated pMST2-T117/low pMST2-T180 is significantly lower than those with low pMST2-T117/high p-MST1-T180 (Figure 5f). Taken together, we conclude that MST2 is a *bona fide* substrate of Akt and that pMST2-T117 could be a prognostic marker in human breast cancer.

**Figure 5:** Akt inhibition of MST2 cellular function depends on the phosphorylation of Thr117. (a) MST2-T117A increases PARP cleavage. HEK293 cells were transfected with indicated plasmids and then immunoblotted with indicated antibodies. (b) Akt inhibits WT-MST2 but not MST2-T117A-induced apoptosis. HEK293 cells were transfected with indicated plasmids. After 36 h of transfection, caspase3/7 activity was measured. The experiment was repeated three times in triplicate. (c) Cell growth curve. Indicated plasmids were introduced into HEK293 cells. Cell number was accounted daily for three days. MST2-T117A significantly inhibited whereas MST2-T117D increased cell growth compared to cells transfected with MST2 or vector alone. (d) Representative breast cancer specimens were lysed and immunoblotted with indicated antibodies. (e) Inverse expression of pMST2-117/Akt-S473 and pMST2-T180 was detected in majority of human breast tumors. (f) Overall survival (OS) in patients with high pMST2-T117/low pMST2-T180 (*n* = 32) versus low pMST2-T117/high pMST2-T180 patients (*n* = 29) was plotted by the Kaplan-Meier method. Statistical comparison of survival between groups with the log-rank statistic analysis suggests that patients whose tumors express pMST2-T117 (+)/pMST2-T180 (−) had poor survival compared to those with pMST2-T117 (−)/pMST2-T180 (+) (*P* = 0.01).

## Discussion

MST1 and MST2 are human homologes of Hippo, however, protein sequence similarity between MST2 and Hippo (63.5%) is higher than that of MST1 versus Hippo (50%). Previous studies have shown that Hippo/MST is autophosphorylated and cleaved by caspases in response to apoptotic stimuli. The cleaved N-terminal kinase domain (e.g., activated MST2) subsequently translocates into the nucleus where it interacts and phosphorylates tumor suppressors Salvador (WW45) and Warts (Lats1/2), which result in inhibition of transcription and/or degradation of DIAPs and cyclin E leading to apoptosis and cell growth arrest [18], [19], [37]. In this study, we demonstrate that IGF1 inhibits MST2 cleavage and activation through the PI3K/Akt pathway. Small molecule inhibitors of PI3K/Akt or depletion of Akt activate MST2. Further, Akt interacts with MST2 and phosphorylates MST2-T117 *in vitro* and *in vivo* leading to inhibition of MST2 cleavage, autophosphorylation and kinase activity. The phosphorylation of Thr117 abrogates MST2 proapoptotic and cell growth-inhibitory function. These results indicate Akt as a key upstream regulator of MST2 and provide a mechanism by which Akt promotes cell survival through direct phosphorylation of MST2 at Thr117 (Figure 6).

**Figure 6:** A diagram represents the regulation of MST2 by IGF1/Akt signal. Under stress conditions, MST2 is activated through caspase-3 cleavage and autophosphorylation-Thr180. The activated/cleaved MST2 translocates to the nucleus and promotes apoptosis. IGF1/Akt inhibits these processes through phosphorylation of MST2-T117.

A previous study has demonstrated that Raf-1 kinase binds to MST2 and prevents its dimerization and autophosphorylation of Thr180, which results in inhibition of MST2 activation and proapoptotic activity [8]. Intriguingly, this regulation is independently of Raf-1 protein kinase activity because kinase-negative Raf-1 also could inhibit MST2 activation and apoptosis [8]. While Akt interacts with MST2, the regulation of MST2 by Akt depends on its kinase activity since constitutively active Akt inhibits whereas dominant-negative Akt induces MST2 activation (Figures 1 and 4). In addition, Akt mediates IGF1 signal towards MST2 and directly phosphorylates Thr117. The phosphorylation of Thr117 is required for Akt inhibition of MST2. Thus, our findings provide the evidence that IGF1/Akt survival signal regulates MST2 through a phosphorylation of Thr117-dependent mechanism.

Our study shows that MST2 possesses an Akt phosphorylation site (^112^RLRNK**T** ^117^) within its N-terminal kinase domain (Figure 1a), which is highly conserved among yeast, *Drosophila*, *Xenopus*, mouse, and human. Moreover, this motif also exists in MST1 (Figure 2b). The Hippo pathway was initially identified in the fly to control organ size. Its core components are evolutionally conserved in mammals. Hippo, Sav, Wts and Mats in the fly are homologous to mammalian MST1/2, WW45, LATS1/2, and Mob1, respectively [38]. Previous studies also showed that the *Drosophila* insulin receptor transduces signals that positively regulate cell and organ growth through its downstream molecule Chico/Dp110/Dakt1 [39], [40]. Overexpression of the *Dakt1* dramatically increases clonal size in wing imaginal disc through an enlargement of the cells [39]. These studies suggest that the crosstalk between Akt and Hippo/MST regulates cell growth and survival and that Akt phosphorylation of MTS2-T117 represents a major regulatory mechanism of the MST2/Hippo pathway among different species.

A previous study showed that Akt phosphorylates Thr387 at C-terminal region of MST1 to abrogate MST1 function [41]. However, Thr387 is not conserved in MST2 and Hippo. As described above, Thr117 of MST2 is conserved in MST1 (Figure 2b). Thus, Akt could regulate both MST1 and MST2 through phosphorylation of the same (e.g., Thr117/Thr120) and different (e.g., Thr387) sites. In addition, it has been shown that full-length and cleaved forms of MST1 and MST2 bind to C-terminal hydrophobic region of Akt and inhibit Akt activation (42), suggesting a negative feedback regulation loop between Akt and MST1/MST2 (Fig. 6). Further investigations are required to define the physiological importance of these Akt phosphorylation sites and feedback regulation between of Akt-MST in knock-in mouse model.

## Supporting Information

Figure S1 MST2-induced apoptosis is inhibited by constitutively active Akt. MCF10A cells were transfected with Flag-MST2 and constitutively active HA-myr-Akt. After 36 h of incubation, cells were subjected to Tunel assay (A) and immunoblotting with indicated antibodies (B).
(2.13 MB TIF)
